# Study on the Countermeasures of Integrating Outdoor Sports into the Development of Health Service Industry in China

**DOI:** 10.1155/2022/1889519

**Published:** 2022-02-12

**Authors:** Dezhi Kong, Jingzhu Sun

**Affiliations:** ^1^Hainan Medical College, Haikou 571199, Hainan, China; ^2^School of Leisure Sports, Xi'an Physical Education University, Xi'an, Shaanxi 710068, China

## Abstract

At present, the exploration and practice of the integration of sports industry, health industry, pension industry, tourism industry, and other related industries are deepening, and outdoor sports have become a way of life for people to entertain, relax, and improve their quality of life. In order to improve the level of people's daily health services and promote the development of sports health services, this paper briefly introduces the development status of outdoor sports in China. Sports health service is an important part of health service industry. It analyzes the development background of sports health service industry from the perspectives of aging population, spreading chronic diseases, and government's attention, sums up the restrictive factors of outdoor sports development, and provides countermeasures and suggestions for the sustainable and healthy development of China's health service industry in the future.

## 1. Introduction

With the improvement of people's living standards and the pursuit of spiritual culture, outdoor sports gradually show its unique market prospect and great economic value. As a result, a number of outdoor products stores have also emerged according to needs, forming a new market potential, with an annual sales of 2 billion Yuan and a participation range of 100 million people. Outdoor sports have quietly become an emerging industry. Outdoor sports have gradually become a sports fashion in China, which also breeds unlimited business opportunities. But, only those who are good at capturing opportunities and dare to innovate can gain something. Therefore, outdoor sporting goods have become a necessity. Taking advantage of the fact that domestic outdoor sports are still in its infancy, it seems to be the best choice to catch this early bus.

Some opinions of the State Council on promoting the development of health service industry clearly defined the connotation and extension of health service industry for the first time, which aims at maintaining and promoting people's physical and mental health, mainly including medical services, health management and promotion, and health insurance and related services, involving supporting industries such as medicines, medical devices, health products, health food, and fitness products [1]. Modern people are often in a state of intense competition and overwork, and there are fewer and fewer opportunities to contact with nature. The characteristics of outdoor sports depend entirely on artificial buildings or the use of natural objects; the project has low requirements on the site [2]. In addition to the huge economic benefits brought by itself, the outdoor sports industry has attracted much attention because of its powerful economic driving role. With more and more people going outdoors, it will further activate the outdoor sports market demand and create greater development space for the outdoor sports industry.

## 2. Understanding of Outdoor Sports

Through consulting the data, it is found that “outdoor sports” in a broad sense refer to all outdoor sports, covering almost all sports. In the narrow sense, outdoor sports refer to sports events that people perform in natural outdoor venues, which can include landscapes and some nonsports facilities or fixed buildings for sports purposes. Outdoor sports are a group of sports events which take the natural environment as the venue (nondedicated venue) and have the nature of adventure or experience adventure. Its main manifestation is to go out of the city, go to nature, and engage in activities with certain risks, challenges, and pertinence on the premise of standardization and safety.

## 3. Development Background of Sports Health Service Industry

### 3.1. The Needs of an Aging Society

China has entered an aging society, and the degree of aging is deepening. According to the 6th National Census, there are 178 million elderly people aged 60 years and over in China, accounting for 13.26% of the total population. Among China's *L* 367 million people, 9.5% are engaged in outdoor sports such as hiking and leisure, and 4.38% are engaged in outdoor sports such as mountaineering, rock climbing, and hiking [3]. With the accelerating pace of urban life, people feel that they are living in a noisy and polluted environment, physically and mentally exhausted, and their physical quality is gradually declining. With the development of outdoor sports, outdoor sports products are gradually known to people. Scientific sports can improve the physical quality of normal old people and achieve the purpose of preventing and treating diseases. The development of outdoor sports presents a diversified and large-scale development trend and also shows the rapid development of outdoor products industry. Therefore, people gradually realized that they should stay away from air pollution and began to pay more and more attention to their physical health.

### 3.2. The State Attaches Great Importance to Them

Outdoor sports are different from indoor sports, which have higher requirements on venues and are greatly influenced by terrain and weather. They not only help people in cities stay away from the hustle and bustle and get close to nature but also have more extensive significance for people to relieve mental stress, enhance their health, and improve their living standards. In recent years, a series of relevant policies have been issued, such as the State Council's opinions on promoting the development of health service industry (2013), the General Office of the State Council's guidance on accelerating the development of sports industry (2010), and the notice on the guidance on accelerating the construction of a social security system and service system for the disabled (2010). By the beginning of the twenty-first century, China's outdoor products industry has taken initial shape and started to develop rapidly [3, 4]. Outdoor sports are different from other strenuous sports, which are not only easy to learn, safe, and effective but also easy to carry out. When applied to the medical field, they can maximize the service benefits, which not only reduces the national investment in medical services but also promotes the health of the masses and relieves the economic burden of society and families.

### 3.3. Chronic Disease Spread

Outdoor sports will affect the development of an industrial chain, including equipment, services, and other industrial categories. However, the scale of outdoor sports activities and competitions in China is relatively small. At present, outdoor activities in China mainly include mountain exploration and mass outdoor activities. In 2011, the World Bank believed that chronic diseases have become the number one health threat in China. If effective strategies are not adopted in time, the number of people over 40 years of age in China suffering from diabetes, cardiovascular diseases, cancer, and chronic respiratory diseases will increase by 2-3 times by 2030. In the field of health talent resources, the management system and mechanism generally lack vitality and have poor management of private market and insufficient protection of basic rights and interests of medical staff. Studies have proved that reasonable physical exercise can effectively control the spread of chronic diseases such as diabetes, hypertension, and obesity and is an economical and efficient treatment [5, 6].

## 4. Restrictive Factors of the Development of Health Service Industry

### 4.1. Restricted by the Level of Economic Development and Income

Outdoor sports are a high-level demand for self-pursuit, which will be restricted by the level of social and economic development and income. Only when people meet the basic needs of food, clothing, housing, and transportation will they consider sports, culture, and entertainment.

In the past, outdoor sports were always associated with young people, mainly from 16 to 35 years of age. However, in the latest survey of outdoor products consumers, the proportion of middle-aged consumers was found to be increasing rapidly, and the proportion of people aged 30–50 years is close to 50%. The specific age distribution is shown in Figure 1.

The noncompetitive and nonexclusive nature of public goods determines that the market is its main supplier. The noncompetitiveness of public goods makes the private market lack power and not able to effectively provide public goods and services. In addition, because public goods are nonexclusive and noncompetitive, their needs or consumption are public or collective. If provided by the market, each consumer will not voluntarily pay for it, but wait for others to buy it and enjoy the benefits it brings. For example, the providers of public sports health services will not get ideal profits because the market cannot efficiently provide noncompetitive and nonexclusive public goods, which is a market failure field in the field of sports health services, and even there is no free market for public sports health services at all. Blind participation in high-risk outdoor sports, which leads to outdoor sports casualties, has become the main cause of accidents.

### 4.2. The Number of Outdoor Sports Activities and Events Is Small, and the Profitability Is Insufficient

Outdoor sports activities and events are the core of outdoor sports industry, but the scale of outdoor sports activities and events in China is relatively small. There is little experience in dealing with sudden accidents, which leads to great potential safety hazards in outdoor sports industry or industry in China, and various accidents occur frequently. Outdoor sports advocate a healthy lifestyle that embraces nature and challenges itself. Compared with developed countries, our country has a weak sense of participation in outdoor sports.

### 4.3. Participants Do Not Know Enough about Outdoor Knowledge

At the initial stage of outdoor sports development, China's outdoor sports industry is still dominated by equipment stores, which mainly represent some foreign brands of equipment. Outdoor sports clubs focus on the practicality of cultivating outdoor sports talents, and they can work in a short time. Outdoor sports have been developed for a short time in China, and many participants have not participated in the training of professional knowledge of outdoor sports. They are not rich in outdoor experience, but only pursue their own fashion and the spirit of going forward bravely, ignoring safety, which makes the danger in the process of sports increase and easily cause accidents.

## 5. Development Strategy of China's Health Service Industry

### 5.1. Establishing and Improving Relevant Laws and Regulations

At present, in the development of sports industry, the legal system is not perfect enough to meet the needs of sports industry in modern commercial society. The legal environment is still in the primary stage and cannot effectively solve various contradictions in the development of sports industry. Therefore, it is necessary to introduce laws and regulations beneficial to standardizing the boundaries of rights subjects, clarifying relevant interest relations and guiding the healthy development of the market in combination with China's actual conditions, timely revise the sports law on the basis of absorbing the operation experience and lessons of existing laws and regulations, and broaden and strengthen the expression scope and strength of the content of the sports industry sector. The formulation and revision of laws and regulations should adapt to the reality of the development of sports industry, be in line with international practices, and pay attention to the protection of individual athletes' interests.

Sound laws and regulations are necessary to ensure the vigorous development of outdoor sports industry. Our government should establish and improve a complete and systematic outdoor sports policy system to create a good platform for the development of outdoor sports in China [7], promote the government to purchase enterprise services, and provide services through the society and the market, and the government pays for services, so that the government and the market can exchange needs and cooperate with each other.

In recent years, with the great concern and support of the party and the government, the Health Qigong Management Center of the State Sports General Administration, the Chinese Health Qigong Association, the International Health Qigong Federation, and other government agencies and nonprofit organizations have played an increasingly important role in the socialization and internationalization of Health Qigong. This activity not only builds a communication platform for health qigong enthusiasts but also creates a social atmosphere of learning and practicing Health Qigong and becomes a brand activity in the national fitness campaign in China (Figure 2).

Compared with physical education classes in schools, outdoor sports lectures in general sense have a relaxed and lively atmosphere and flexible and diverse teaching methods and are also popular among students and the public. Outdoor sports club is one of the main ways to organize outdoor activities, and the transmission of activity information is mainly through websites, so outdoor clubs and website forums can be used to develop potential customers.

### 5.2. Marketing Strategy of Promoting Product Sales by Club Activities

Outdoor sports clubs are organizations that provide outdoor sports enthusiasts with various forms of services such as organizing activities, organizing various competitions, providing training, and conducting lectures. From the perspective of outdoor sports itself, as a branch of sports industry, it has great similarities with health industry, and the common purpose is to serve health. Therefore, the basic form of training outdoor sports talents can be to train all kinds of outdoor sports talents in the form of teachers with apprentices (that is, to let qualified outdoor sports professionals with long experience lead 2-3 students) or short-term training courses. Professional and systematic theoretical guidance should be given to students, and outdoor practical courses such as rock climbing, downhill, and crossing should be offered to enable students to deal with emergencies, improve their abilities, and challenge themselves in real outdoor situations.

### 5.3. Concising the Professional Team and Providing the Team Foundation for the Development of Outdoor Sports Health Service Industry

Having excellent and professional talents is the foundation and guarantee for the development of health service industry. Because the number of outdoor sports clubs is relatively small, outdoor sports enthusiasts are widely distributed, and direct sales promotion is not effective. In today's society, the Internet is increasingly becoming an indispensable communication medium for people, and it can be said to be a very useful way to spread outdoor sports. Outdoor sports majors or outdoor sports courses can be opened in sports colleges and universities, and sports experts and outdoor experienced talents can be organized to prepare outdoor sports professional teaching materials, such as introduction to outdoor sports and outdoor self-help. Investing in R&D and promoting the transformation of scientific and technological achievements in sports health services can not only ensure the sustainable development of enterprises but also greatly promote the development and maturity of China's health service industry.

### 5.4. Management Marketing Team Building

The construction of the management and marketing team directly determines the survival of the company. As a new service, customer positioning, product design, market development, media operation, service refinement, enterprise visibility, and reputation are the keys to determine whether an enterprise can make a profit. The core purpose of establishing the internal training system of the enterprise is to improve the work skills and performance of employees and the overall performance of the company. This requires us to clarify the responsibilities of each department for training, supervise training, evaluate, and feed back the training effect when establishing the internal training system of the enterprise. The core purpose of establishing the internal training system of the enterprise is to improve the work skills and performance of employees and the overall performance of the company. This requires us to clarify the responsibilities of each department for training, supervise training, evaluate, and feed back the training effect when establishing the internal training system of the enterprise. The education and training system of outdoor sports professional knowledge and skills should be improved, and targeted professional guidance should be provided to club managers, event organizers, and outdoor sports participants who have been engaged in outdoor work. The broadcast of TV programs related to outdoor sports will also play a very positive role in guiding and popularizing outdoor sports. You can also use the network to build an online platform, establish technical and business cooperation with sports and medical and other application software, promote and publicize outdoor sports, and change some prejudice of young people against outdoor sports. On the Internet, we can establish a platform for people who love outdoor sports to learn and communicate by creating related online post bars and setting up special outdoor sports websites.

## 6. Conclusions

If the sports health service industry wants to have a great development, it must overcome its own shortcomings and strengthen its efforts in product design, marketing management, and talent development. The sports health service industry will have a great development. People's diversified sports and health needs are facing obvious supply side deficiencies, and the sports consumption mode is gradually changing from physical consumption to participatory consumption. Through the analysis of the development status of outdoor sports in China, it is found that outdoor sports in China develop rapidly, while the popularization of outdoor sports knowledge is relatively backward, which is not conducive to the healthy development of outdoor sports and needs to be further popularized. The national traditional sports industry represented by outdoor sports is facing great development opportunities. Therefore, in the future, the research on sports healthcare services in China will continue to increase.

## Figures and Tables

**Figure 1:** Consumption proportion of outdoor products in different age groups.

**Figure 2:** The increasing trend of the number of people practicing Health Qigong in China from 2011 to 2020.

## Data Availability

The data used to support the findings of this study are included within the article.
